# Immunomodulatory Effects of Combined Ethanol Extracts of *Curcuma mangga* and *Picria fel-terrae* on Cellular- and Humoral-Mediated Immunity in Wistar Rats and Mice

**DOI:** 10.1155/2022/1791165

**Published:** 2022-09-20

**Authors:** Yuandani Yuandani, Ibrahim Jantan, Lia Laila, Marianne Marianne, Abdi Wira Septama, Ngagami Lintang, Putri Almadani, Friti, Syarifah A'ini

**Affiliations:** ^1^Department of Pharmacology, Faculty of Pharmacy, Universitas Sumatera Utara, Medan, Indonesia; ^2^Centre of Excellence for Chitosan and Advanced Materials, Universitas Sumatera Utara, Medan, Indonesia; ^3^Institute of Systems Biology, Universiti Kebangsaan Malaysia (UKM), Bangi, Selangor, Malaysia; ^4^Department of Pharmaceutical Technology, Faculty of Pharmacy, Universitas Sumatera Utara, Medan, Indonesia; ^5^Research Center for Pharmaceutical Ingredients and Traditional Medicine, National Research and Innovation Agency (BRIN), Kawasan PUSPIPTEK Serpong, Tangerang Selatan, Banten, Indonesia

## Abstract

Previous studies have shown that the extracts of *Curcuma mangga* Valeton & Zijp rhizomes and *Picria fel-terrae* Lour. leaves could modulate cellular- and humoral-mediated immunity in macrophages and animal models. In the present study, the immunomodulatory effects of combined ethanol extracts of *C. mangga* rhizomes and *P. fel-terrae* leaves were investigated on cellular- and humoral-mediated immunity in Wistar rats and mice. The phytochemical constituents of the ethanol extracts of *C. mangga* and *P. fel-terrae*, and combined extracts were analyzed by high-performance liquid chromatography-tandem mass spectrometry (HPLC-MS/MS). Mice were orally administered with combined extracts of *C. mangga* and *P. fel-terrae* (1 : 1) at doses of 25, 50, and 100 mg/kg·bw for 7 days, and the carbon clearance method was used to investigate their phagocytosis activity. Wistar rats were treated orally with the combined extracts 72 h prior to sensitization with *Staphylococcus aureus* and continued for 14 days. The effect of extracts on delayed-type hypersensitivity (DTH) response was determined by the paw edema method, while the effects on antibody (IgG and IgM) and interleukin-2 (IL-2) production were analyzed using enzyme-linked immunosorbent assay (ELISA). Picfeltarraenin VI and ferruginol were the major components in the extracts of *P. fel-terrae* and *C. mangga*, respectively. The combined extracts at 1 : 1 ratio demonstrated a dose-dependent stimulation of both cellular- and humoral-mediated immunity in both animal models. The combined extracts displayed the strongest stimulation on DTH response and phagocytosis activity at 100 mg/kg·bw, which were comparable with those of the positive control, levamisole. IgG and IgM production and IL-2 release were also stimulated after treatment with extracts. The combined extracts of *C. mangga* and *P. fel-terrae* possess strong stimulatory activities on cellular- and humoral-mediated immunity and may be developed as a potential nutraceutical for the modulation of immune responses.

## 1. Introduction

The human defense system against pathogens consists of various components that are interconnected in a highly coordinated network [1]. Phagocytes play a necessary role in the nonspecific immune system. The complement system of the humoral component is essential in regulating innate immune response and strengthening the phagocytosis ability of phagocytes. It can be activated through several pathways such as the alternative pathway, which is activated by a number of microorganisms spontaneously [2]. This activation generates peptide fragments, which have several functions that include opsonization of microbes, the attraction of phagocytes to sites of infection, and release of further inflammatory mediators (e.g., histamine and leukotriene) [3]. Meanwhile, lymphocytes are the main cellular component in adaptive immunity. The regulatory functions are mediated mainly by T helper (Th) cells that stimulate B cells to produce antibodies [4].

In humans, the antibody can be divided into five classes that differ from each other in the heavy chains of immunoglobulin molecules (*α*, *δ*, *ε*, *γ*, and *μ*); these include immunoglobulin A (IgA), IgD, IgE, IgG, and IgM [5]. IgG is the most predominant immunoglobulin in the serum and the most important antibody in serosal immunity. It has a high affinity to the antigen, and IgG-antigen complexes can be recognized by complement factors and by Fc receptors on the surface of phagocytes. In both cases, IgG binding leads to the elimination of antigen-bearing cells [6]. IgM is the first antibody produced by the fetus and is also the first antibody to respond when presented with a new antigen challenge. In the primary response against a new antigen, the appearance of IgM in the blood precedes that of IgG. The production of IgM decreases when the production of IgG increases [7].

The signaling process between cells during immune responses is facilitated by cytokines [3]. Cytokines can be derived from any cells such as lymphocytes and have been shown to be involved in autocrine, paracrine, and endocrine signaling as immunomodulatory agents. Interleukin-2 (IL-2) acts as paracrine signals to regulate the development of mature T cells [8]. Moreover, IgG and IgM production from activated B lymphocytes is facilitated by IL-4 [9]. All those cells and soluble products are interrelated and act to fight invading organisms. However, the dysfunction of immune response may cause various diseases, such as ulcerative colitis (UC), psoriasis, rheumatoid arthritis (RA), and immunodeficiency disorders. Thus, the modulation of immune responses is required for the treatment of those diseases [10].

Traditional herbs have been used as an alternative medicine to treat various diseases including immune-related diseases for many years ago. The extracts of many medicinal plants such as *Camellia sinensis*, *Gynura segetum*, *Aglaonema hookerianum, Lannea coromandelica*, *Curcuma mangga*, and *Picria fel-terrae,* and their bioactive secondary metabolites have been investigated for their pharmacological activities [11–17]. *Curcuma mangga* Valeton & Zijp. rhizomes are utilized in traditional medicine to cure various diseases such as in the treatment of fever, stomach disorders, and cancer [18]. *C. mangga* was found to be rich in flavonoids, glycosides, terpenoids, and steroids [16]. The inhibitory effects of demethoxycurcumin, bisdemethoxycurcumin, (E)-15,15-diethoxylabda-8(17),12-dien-16-al, and 15,16-bisnorlabda-8(17),11-dien-13-one isolated from *C. mangga* on production of prostaglandin E2 and nitric oxide (NO) in RAW 264.7 cells have been reported previously [19]. The analgesic activity of *C. mangga* extract and fractions on nociceptive responses was evaluated using a hot plate, writhing, and formalin tests in mice, while their anti-inflammatory activity was determined using inflammatory models of croton oil-induced mouse ear edema and carrageenan-induced rat paw edema [20]. The immunomodulatory activities of *C. mangga* rhizome extract on phagocytosis, cytokine gene expression, antibody production, and DTH response in macrophages and different animal models have been reported by us previously [16, 21, 22]. The engulfment of mouse leukocytes was enhanced by the immunostimulatory effect of various solvent extracts of *C. mangga* [22]. In another study, the *C. mangga* ethanol extract displayed an increase in phagocytosis ability dose-dependently, with a higher phagocytic index than that of negative control, indicating its strong immunostimulatory activity [16]. It was shown that the extract downregulated IL-6, IL-1*β*, and tumor necrosis factor-*α* (TNF-*α*) gene expression as compared to the negative control in lipopolysaccharide(LPS)-induced RAW 264.7 cells. The extract increased IgG production in cyclophosphamide-induced *Salmonella typhimurium*-infected rats, which was comparable with that of levamisole as a positive control. However, the extract displayed the inhibition of production of IL-4 dose-dependently in normal and cyclophosphamide-induced immunosuppressed rats [22]. It was also shown that the extract increased the rat paw volume after infected with *S. typhimurium,* enhancing the DTH response of immunosuppressed rats [22]. Toxicological investigation into *C. mangga* rhizome extract in Wistar rats indicated that it was nontoxic with an LD_50_ value of greater than 5000 mg/kg·bw. In addition, it was shown that pregnant animals orally treated with *C. mangga* were safe without uterus and fetal toxicities at certain doses [23].

*Picria fel-terrae* Lour. has been used traditionally to treat cough, stomach aches, asthma, and inflammation. A previous study has found that *P. fel-terrae* contained saponins, glycosides, saponins, and terpenoids [24]. *P. fel-terrae* was reported in a previous study to be able to regulate NO production from LPS-induced RAW 264.7 cells. It was shown that the *n*-hexane extract of *P. fel-terrae* exhibited the strongest inhibition on NO production compared with the ethanol and ethyl acetate extracts of the plant [17]. Amongst the extracts tested, the ethyl acetate extract of *P. fel-terrae* at 200 mg/kg·bw exhibited the strongest phagocytosis activity in white male mice using the carbon clearance method [25]. Recently, it was revealed that the *P. fel-terrae* ethanol extract exhibited an immunomodulatory effect by increasing TCD4+ and TCD8+ levels in doxorubicin-induced immunosuppressed rats [26]. Investigation into subchronic toxicity of the *P. fel-terrae* extract in Wistar rats indicated that it was nontoxic on long-term use [24].

According to the previous studies mentioned above, the individual extracts of *Curcuma mangga* and *Picria fel-terrae* have immunomodulatory activities [16, 17, 21, 22, 25, 26]. The results of these studies indicate that the extracts of the plants could individually modulate the cellular- and humoral-mediated immunity in macrophages and animal models. The novelty of the present study is on the determination of immunomodulating effects of the combined extracts of *C. mangga* and *P. fel-terrae* on cellular- and humoral-mediated immunity in Wistar rats and mice. This is the first report on the immunomodulating effects of combined extracts of *C. mangga* and *P. fel-terrae* in modulating cellular- and humoral-mediated immunity in both animal models. In this paper, we report on the immunomodulatory effects of combined extracts of *C. mangga* and *P. fel-terrae* on phagocytosis activity in mice, as well as DTH response, and antibody and cytokine production from *Staphylococcus aureus-*infected Wistar rats. The major components of the combined extracts and the individual extract were analyzed by high-performance liquid chromatography-tandem mass spectrometry (HPLC-MS/MS).

## 2. Materials and Methods

### 2.1. Plant Materials and Preparation of Plant Extracts

The rhizomes of *C. mangga* and whole plant (without root) of *P. fel-terrae* were obtained from North Sumatera Province, Indonesia. The plant samples were authenticated by a botanist, and voucher specimens were deposited at the Herbarium Medanese (MEDA), Universitas Sumatera Utara (USU), Medan, Indonesia, with voucher number of 6179/MEDA/2021 and 6180/MEDA/2021 for *C. mangga* and *P. fel-terrae*, respectively. Briefly, the plant materials were dried in a drying cabinet at 40–50°C. Then, the dried *C. mangga* rhizomes (700 g) were ground into powder and soaked with absolute ethanol [1 : 10 (w/v)] in a closed glass container at room temperature. The mixture was frequently stirred, and the solvent was filtered through Whatman No. 1 filter paper (Whatman, England). The solvent was then removed under reduced pressure using a rotary evaporator at 45–50°C to obtain the crude extract. The same procedure was applied to *P. fel-terrae* to obtain *P. fel-terrae* extract [22].

### 2.2. Antigen Preparation

One mL aliquot of *Staphylococcus aureus* (ATCC 25923), procured from the American Type Culture Collection (ATCC, USA) was diluted with a nutrient broth to obtain a cell concentration of 1 × 10^8^ cells/mL. The cell concentration was calculated according to the turbidimetric method using a spectrophotometer with an optical density of 530 nm as stated in Indonesian Pharmacopoeia [27]. The mixture was centrifuged at 25°C for 10 min at 10,000 rpm. The cells were separated and then washed with 1 mL of phosphate buffer saline (PBS) (Sigma, USA) [22].

### 2.3. LC-MS/MS Analysis of Individual Extract and Combined Extracts of *C. mangga* and *P. fel-terrae*

The extracts were subjected to LC-MS/MS analysis on C18 column (Waters Acquity BEH C18 50 mm × 2.1 mm). Separation was performed with a sample injection volume of 1 *μ*L and gradient elution at a flow rate of 0.3 mL/min at a column temperature of 40°C, using a gradient method containing solvents A (0.1% formic acid) and B (100% acetonitrile) as eluents with a total running time of 17 min. The elution began with 5% B (0-1 min), 100% B (1–14 min), and finally 5% B (14–17 min). High-resolution mass spectrometry was carried out using a Xevo G2-XS QTof (Waters), with an ESI-positive ionization. The mass range was at 100–1200 *m*/*z*. The accurate mass data of the molecular ions, provided by the TOF analyzer, were processed by Waters UNIFI 1.8.1 Scientific Information System Release Note 716004598, Revision B. The compounds were identified by comparing their mass fragmentation patterns with respective standards in the mass spectral library database.

### 2.4. Animals

A total of 50 male Wistar rats (120–200 g; 2-3 months old) and 25 mice (20–30 g; 2-3 months old) were used. The animals were supplied by the Animal Breeding Laboratory, Universitas Sumatera Utara. The principles for animal care and use by the National Agency of Drug and Food Control (NA-DFC) were followed to handle the animals. Acclimatization of test animals was carried out by placing mice and rats in plastic cages with standard environmental conditions for 7–14 days at room temperature with adequate ventilation before the experiment. The animals were provided with a standard pellet diet and water ad libitum.

### 2.5. Delayed-Type Hypersensitivity (DTH) Response

The effect of extracts on DTH response was determined by measuring the change in paw volume in rats as described previously [22]. A preliminary study was performed to select the combination ratio of *C. mangga* and *P. fel-terrae* that produced the strongest stimulation. The five Wistar rats of each group were administered with the combined extracts at three different combination ratios of *C. mangga* and *P. fel-terrae*, i.e., 1 : 1, 1 : 3, and 3 : 1. Of all the ratios, the combined extracts of *C. mangga* and *P. fel-terrae* at 1 : 1 ratio demonstrated the strongest stimulation on cellular immunity. The combined extracts at 1 : 1 ratio were further used to demonstrate the effect of the extracts on DTH response at various concentrations. Briefly, the rats were sensitized with *S. aureus* (1 × 10^8^ cells/mL) by intraperitoneal injection followed 72 h later by administration of the combined extracts (1 : 1) at doses of 25, 50, and 100 mg/kg·bw and continued for 14 days. The negative control contained 0.5% sodium carboxymethylcellulose (CMC Na) only, while Imboost® (32.5 mg/kg·bw) was used as the positive control. On day 14, a Plethysmometer (Ugo Basile, Italy) was used to measure the hind paw volume of rats. The animals were then challenged by a subcutaneous injection of *S. aureus* in their hind paws, and 24 h later, the mean increase in paw volume was measured.

### 2.6. Phagocytosis Assay

A carbon clearance method was used to determine the effect of combined extracts of *C. mangga* and *P. fel-terrae* on phagocytosis ability [28]. Briefly, twenty-five mice (five mice of each group) were administered with the combined extracts of *C. mangga* and *P. fel-terrae* in the equal ratio (1 : 1) at doses of 25, 50, and 100 mg/kg·bw for 7 days. The vehicle 0.5% CMC Na and Imboost® (32.5 mg/kg·bw) were used as negative and positive control, respectively. All the animals were administered with a dispersion of China ink (0.1 mL per 10 g) by intravenous injection *via* tail vein on day 8. Blood samples (25 *μ*L) were then collected at an interval of 5, 10, 15, and 20 min from each animal. The erythrocytes were lysed by adding 4 mL of 1% acetic acid to the blood samples to lyse the erythrocytes. A Thermo Scientific microplate reader (Thermo Fisher Scientific, USA) was used to measure the absorbance of the supernatants at 640.5 nm. Finally, 12 h after blood collection, the animals were humanely euthanized by cervical dislocation and their spleens and livers were discarded. The following equations were used to calculate the rate of carbon clearance and phagocytic index.

(1) $$\begin{array}{c} \text{Rate of carbon clearance}\left(K\right)=\frac{\text{LogOD}5-\text{logOD}20}{t2-t1}, \end{array}$$

(2) $$\begin{array}{c} \text{Phagocytic index}\left(\alpha \right)=\frac{K^{1/3}\times \text{animal body wt}}{\text{Liver wt}+\text{spleen wt}}, \end{array}$$

where OD5 is the log absorbance of blood at 5 min; OD20 is log absorbance of blood at 20 min; *t*2 is the last time point of blood collection; and *t*1 is the first time point of blood collection.

### 2.7. Immunomodulatory Assay on Antibody and Cytokine Production

The effects of extracts on antibody and cytokine production were evaluated as described previously [22]. The five Wistar rats of each group were similarly sensitized with *S. aureus* and then treated with the combined extracts of *C. mangga* and *P. fel-terrae* at various concentrations, as described above in the procedure for DTH response. Levamisole (25 mg/kg·bw) was used as a positive control. Blood was collected on day 15, and the serum was used for the determination of IgG, IgM, and IL-2 using ELISA kits procured from LABISKOMA (Korea).

### 2.8. Statistical Analysis

The data were presented as mean and standard error mean (SEM) and were statistically analyzed by a one-way analysis of variance (ANOVA), followed by the post hoc Tukey test. Differences were considered significant when *P* values were less than 0.05. The combination index was determined using the CompuSyn software.

## 3. Results

### 3.1. LC-MS/MS Analyses of *C. mangga*, *P. fel-terrae*, and Combined Extracts

In this current study, 78.91 g (11.27%) and 56.71 g (8.1%) of *C. mangga* and *P. fel-terrae* extracts were obtained, respectively. LCMS/MS analysis of *C. mangga* revealed the presence of ferruginol, (E)-labda-8(17),12-diene-15,16-dial, saurufuran B, and sugiol with ferruginol as the most abundant compound with a retention time (RT) of 10.95 min (Figure 1(a)). Analysis of chromatogram of *P. fel-terrae* extract led to the identification of picfeltarraenin VI, abrusoside A, skimmin, and trichosanic acid (Table 1). Picfeltarraenin VI (picfeltarraegenin I 3-O-*β*-d-xylopyranoside) at the RT of 5.51 min was identified as the most prominent compound (Figure 1(b)). However, only some compounds could be identified in the combined extracts of *C. mangga* and *P. fel-terrae,* namely, (E)-labda-8(17),12-diene-15,16-dial, abrusoside A, ferruginol, picfeltarraenin VI, and sugiol. Skimmin and trichosanic acid, which were identified in *P. fel-terrae* extract, could not be identified in the combined extracts due to overlapping of peaks (Figure 1(c)). The major compounds identified in the combined extracts were ferruginol and picfeltarraenin VI with the former as the most abundant compound. The chemical structures of compounds identified in the extracts are shown in Figure 2.

### 3.2. Delayed-Type Hypersensitivity (DTH) Response

A preliminary study on the effect of different combination ratios of the plant extracts on DTH response indicated that the combined extracts of *C. mangga* and *P. fel-terrae* at 1 : 1 ratio demonstrated the strongest stimulation of cellular immunity. The paw volume of 1.44 ± 0.051 mL exhibited by the 1 : 1 ratio combination was comparable to that of the positive control, levamisole (1.52 ± 0.03 mL) (Table 2).  Figure 3 shows that the effect of the combined extracts of plants (1 : 1) on DTH response was dose-dependent. The paw thickness was higher than that of negative control (*P* < 0.05), indicating that they were enhancing cell-mediated immunity. The combination index that was determined using CompuSyn revealed that it has strong synergistic activity with the combination index (CI) of 0.26706.

### 3.3. Phagocytosis Assay

Table 3 shows that the rate of carbon elimination after treatment with different doses (25, 50, and 100 mg/kg·bw) of the combined extracts of *C. mangga* and *P. fel-terrae* was higher than that of negative control (*P* < 0.05), indicating that they were enhancing the percentage of carbon engulfment and thus inducing the phagocytic cells. The combined extracts of the plants dose-dependently stimulated the carbon ingestion. The combined extracts showed the highest stimulation at a dose of 100 mg/kg·bw, exhibiting a phagocytic index of 5.44 ± 0.08, which was comparable to that of Imboost®, the positive control, with a phagocytic index of 6.39 ± 0.03 (Figure 4).

### 3.4. Immunomodulatory Assay on Antibody and Cytokine Production

The combined extracts of *C. mangga* and *P. fel-terrae* upregulated the production of IgM and IgG from *S. aureus-*infected rats dose-dependently (Table 4). At the highest dose of 100 mg/kg·bw, the extracts stimulated IgM and IgG production to 1.47 ± 0.08 and 1.60 ± 0.06 ng/mL, respectively, which were higher than those stimulated by levamisole (25 mg/kg·bw). Moreover, the extracts were able to enhance the production of IgM and IgG as compared to the negative control (*P* < 0.05). Similarly, the extracts also dose-dependently stimulated production of IL-2 as shown in Table 4. The extracts at the highest dose of 100 mg/kg·bw demonstrated the strongest stimulation, exhibiting a value of 20.34 ± 3.18 ng/mL, which was higher than that of levamisole (18.70 ± 2.09 ng/mL).

## 4. Discussion

The HPLC-MS/MS analysis indicated the presence of picfeltarraenin VI and ferruginol as the major components in the extracts of *P. fel-terrae* and *C. mangga*, respectively. Investigation into the effect of combined extracts on immune response was initiated by determining the combination ratio of *C. mangga* and *P. fel-terrae* that produced the strongest stimulation. Of all the ratios, the combined extracts of *C. mangga* and *P. fel-terrae* at 1 : 1 ratio showed the highest stimulation on DTH response. Furthermore, the combined extracts at ratio 1 : 1 at the doses of 25, 50, and 100 mg/kg·bw were investigated for their effects on DTH response, phagocytosis activity, and immunoglobulin and cytokine production. The combination of *C. mangga* and *P. fel-terrae* extracts was able to enhance the DTH response. DTH is a cellular-mediated immunity that is mediated by the stimulation of T lymphocytes and followed by the release of cytokines. In turn, cytokines stimulate the macrophages to initiate inflammation as a defensive response, which is indicated by paw edema formation [3]. The stimulatory activity of the herbal combination, especially at the dose of 100 mg/kg·bw on DTH response, was higher (paw volume 1.44 ± 0.11 mL) when compared to *C. mangga* extract alone (paw volume: 0.88 ± 0.03 mL) as reported in a study by Yuandani et al. [29]. There might be a strong synergistic effect of the herbal combination to stimulate DTH response. This result was supported by the combination index value (CI: 0.26706), which indicates the strong synergistic activity.

Phagocytosis is the main cellular innate immune response to eradicate pathogens. The innate immune system detects invading pathogens through several pattern recognition receptors (PRRs), which recognize pathogen-associated molecular patterns (PAMPs) on the pathogens. Engagement of PRR with infectious agents initiates phagocytosis [30]. Phagocytosis involves ingestion of particulate ligands, often multiple and large particles with a size exceeding 1 *μ*m. This phenomenon accomplishes two important immune functions, i.e., as an innate immune effector and a bridge between the nonspecific and specific immune responses. The enhancement of phagocytosis ability to eliminate pathogens markedly enhances the host defense to protect the body from invading organism [31]. The effect of combined extracts of *C. mangga* and *P. fel-terrae* on phagocytosis activity was evaluated by the carbon clearance method. The increment of phagocytosis activity of mouse leukocytes was presented by the increased clearance rate of carbon particles from the bloodstream. The activity of the combined extracts was comparable to that of Imboost® as a positive control. Imboost®, a marketed herbal formulation to enhance the immune system, contains *Echinacea purpurea* that has been reported to have stimulatory activity on cytokine release from macrophages [32]. Interestingly, at the dose of 100 mg/kg·bw, the combined extracts of *C. mangga* and *P. fel-terrae* showed a phagocytic index of 5.44 ± 0.08, which was higher than that of *C. mangga* extract alone [16]. The results indicate that the herbal combination was more effective than the single extract in stimulating phagocytosis ability.

The immunomodulatory effects of the combined extracts on immunoglobulin and cytokine production were investigated using *S. aureus*-infected Wistar rats as the animal model. In the present study, the rat defense against *S. aureus* was initiated by the innate arm of immune response. Through innate immune recognition, inflammatory cascades were initiated, which include leukocyte chemotaxis towards the site of infection, activation of antimicrobial mechanisms, then induction of the specific immune response [33].

The combined extracts of *C. mangga* and *P. fel-terrae* also enhanced IL-2 release. IL-2 is involved in B- and T-lymphocyte proliferation and differentiation, as well as plays a necessary role in stimulating IgG1 and IgE isotype production [34, 35]. In this study, the combined extracts enhanced the production of IgM, IgG, and IL-2 in *S. aureus*-infected Wistar rats. IL-2 is an essential cytokine in T-lymphocyte proliferation. The antibody is known to be produced from B lymphocytes through T-dependent or T-independent pathways. Thus, the increase in the production of IgG and IgM by the combined extracts might be due to the activation of T-dependent immune response [36]. The results indicate the ability of combined extracts to stimulate lymphocyte proliferation and subsequently enhance antibody production.

Polyherbal formulations are prepared using combined extracts of medicinal plants to enhance their desired effects or to produce synergistic effects. The immunostimulatory effects of combined extracts of *C. mangga* and *P. fel-terrae* in modulating cellular- and humoral-mediated immunity in both animal models may suggest that the stimulatory effect was due to positive interactions between bioactive components of both plants. The strong immunostimulatory effect of combined extracts of *C. mangga* and *P. fel-terrae* indicates their potential to be developed into a potent nutraceutical for the modulation of immune responses for the prevention and treatment of various diseases, such as immunodeficiency and cancer. Several studies have reported the adverse events of immunotherapy of biologic agents in cancer [37]. Thus, the combined extracts of the plants have great potential to be further developed into a safe and effective agent for the prevention and treatment of cancer. However, the molecular mechanisms underlying the synergistic effects have to be investigated to provide a better understanding of the immunostimulatory effect of the combined extracts. There are many studies on the synergistic effects of combined extracts of various medicinal plants. The neuroprotective- and cognitive-enhancing effects of the combined extracts of *Zingiber officinale* and *Cyperus rotundus* on the improvement of age-related dementia in rats with AF64A-induced memory deficits have been reported [38]. The synergistic anti-inflammatory activity of *Cassia fistula* and *Solanum xanthocarpum* has also been documented [39].

## 5. Conclusions

The combined extracts of *C. mangga* and *P. fel-terrae* were able to enhance the immune response in cellular- and humoral-mediated immunity in mice and rats. The extracts strongly enhanced phagocytosis ability in mice, and stimulated DTH response, IL-2 release, and antibody (IgM and IgG) production in *S. aureus*-infected rats. Moreover, the combined extracts revealed stronger immunostimulatory activity on DTH response and phagocytosis ability than the individual extract when tested under the similar condition as reported in previous studies. The immunostimulatory activity of the extracts could be due mainly to picfeltarraenin VI and ferruginol although the contribution of the other constituents of the plant extracts should not be excluded. The stimulatory effect might be due to positive interactions between the bioactive components of both plants. The results revealed that the combined extracts of *C. mangga* and *P. fel-terrae* have potential to be developed into a potent nutraceutical for the modulation of immune responses. However, their mechanisms of action in different lineages of immune responses require further elucidation.

## Figures and Tables

**Figure 1:** LC-MS/MS chromatogram of (a) *C. mangga* rhizome extract, (b) *P. fel-terrae* herb extract, and (c) combined extracts of *C. mangga* and *P. fel-terrae*.

**Figure 2:** Chemical structures of compounds identified in *C. mangga* and *P. fel-terrae*.

**Figure 3:** Effect of combined extracts of *C. mangga* and *P. fel-terrae* on delayed-type hypersensitivity (DTH) response in *S. aureus-*infected rats (mean ± SEM; ^*∗*^*P* < 0.05 is significant to respective control).

**Figure 4:** Effect of combined extracts of *C. mangga* and *P. fel-terrae* on a phagocytic index in *S. aureus-*infected rats (mean ± SEM; ^*∗*^*P* < 0.05 is significant to respective control).

**Table 1:** Retention times, MS fragments of the major compounds present in the ethanol extracts of *C. mangga* and *P. fel-terrae,* and their combined extracts.

Samples	RT	Observed *m*/*z*	MS^2^ fragmentation ions	Tentative identification
*P. fel-terrae* extract	5.1	647	485, 467, 449, 309, 291	Abrusoside A
	5.51	617	485, 467, 449, 309, 291, 175	Picfeltarraenin VI
	3.33	325	309, 287, 181, 163,	Skimmin
	9.27	279	261, 243, 209	Trichosanic acid

*C. mangga* extract	9.27	303	285, 267, 241, 217	(E)-labda-8(17),12-diene-15,16-dial
	10.95	285	267, 241, 187, 139	Ferruginol
	8.84	317	301, 185, 128	Saurufuran B
	10.1	301	255, 185, 163	Sugiol

Combined extracts of *C. mangga* and *P. fel-terrae*	9.28	303	285, 267, 241, 217	(E)-labda-8(17),12-diene-15,16-dial
	5.1	647	485, 467, 449, 309, 291	Abrusoside A
	10.95	285	267, 241, 187, 139	Ferruginol
	5.51	617	485, 467, 449, 309, 291, 175	Picfeltarraenin VI
	10.1	301	255, 185, 163	Sugiol

**Table 2:** Effect of various combination ratios of *C. mangga* and *P. fel-terrae* on delayed-type hypersensitivity (DTH) response in *Staphylococcus aureus-*infected rats.

No.	Samples	Paw volume (mL)
1	0.5% CMC Na	0.320 ± 0.037
2	*C. mangga* 100 mg/kg·bw + *P. fel-terrae* 100 mg/kg·bw (1 : 1)	1.440 ± 0.051^*∗*^
3	*C. mangga* 50 mg/kg·bw + *P. fel-terrae* 150 mg/kg·bw (1 : 3)	1.180 ± 0.081^*∗*^
4	*C. mangga* 150 mg/kg·bw + *P. fel-terrae* 50 mg/kg·bw (3 : 1)	1.220 ± 0.059^*∗*^
5	Levamisole 25 mg/kg·bw	1.520 ± 0.030^*∗*^

^*∗*^ *P* < 0.05 is significant to respective control; data: mean ± SEM.

**Table 3:** Effect of combined extracts of *C. mangga* and *P. fel-terrae* on carbon clearance rate.

No	Samples	Carbon clearance rate
1	CMC Na (0.5%)	0.0151 ± 0.0002
2	Imboost® (32.5 mg/kg·bw)	0.0560 ± 0.0058^*∗*^
3	Combined extracts (25 mg/kg·bw)	0.0311 ± 0.0002^*∗*^
4	Combined extracts (50 mg/kg·bw)	0.0301 ± 0.0001^*∗*^
5	Combined extracts (100 mg/kg·bw)	0.0455 ± 0.0005^*∗*^

^*∗*^ *P* < 0.05 is significant to respective control; data: mean ± SEM.

**Table 4:** Effect of combined extracts of *C. mangga* and *P. fel-terrae* on antibody and cytokine production from *Staphylococcus aureus*-infected rats.

No	Samples	Antibody and cytokine levels (ng/mL)		
		IgM	IgG	IL-2
1	0.5% CMC Na	0.63 ± 0.16	0.81 ± 0.17	8.67 ± 0.34
2	Levamisole (25 mg/kg·bw)	1.38 ± 0.05^*∗*^	1.52 ± 0.09^*∗*^	18.70 ± 0.94^*∗*^
3	Combined extracts (25 mg/kg·bw)	1.28 ± 0.04^*∗*^	1.36 ± 0.05^*∗*^	13.63 ± 1.08^*∗*^
4	Combined extracts (50 mg/kg·bw)	1.32 ± 0.06^*∗*^	1.48 ± 0.04^*∗*^	16.84 ± 1.04^*∗*^
5	Combined extracts (100 mg/kg·bw)	1.47 ± 0.08^*∗*^	1.60 ± 0.06^*∗*^	20.34 ± 1.42^*∗*^

^*∗*^ *P* < 0.05 is significant to respective control; data: mean ± SEM.

## Data Availability

All data generated to support the results of this study are available from the corresponding author on reasonable request.
